# Intracoronary Ultrasound Imaging Combined with Traditional Chinese Medicine Nursing Applied in the Treatment of Coronary Heart Disease Patients with Phlegm and Blood Stasis Syndrome

**DOI:** 10.1155/2022/2820851

**Published:** 2022-08-21

**Authors:** Hui Zeng, Chunmian Guo, Yan Yang, Xia Chu, Yanru Shi

**Affiliations:** ^1^Department of Traditional Chinese Medicine, First Affiliated Hospital of Air Force Military University (Xijing Hospital), Xi'an 710032, Shaanxi, China; ^2^Department of Cardiology, First Affiliated Hospital of Air Force Military University (Xijing Hospital), Xi'an 710032, Shaanxi, China; ^3^Department of General Practice, First Affiliated Hospital of Air Force Military University (Xijing Hospital), Xi'an 710032, Shaanxi, China; ^4^Department of Psychiatry, First Affiliated Hospital of Air Force Military University (Xijing Hospital), Xi'an 710032, Shaanxi, China

## Abstract

This study was to explore the effect of traditional Chinese medicine (TCM) nursing intervention based on intracoronary ultrasound imaging on patients with coronary heart disease (CHD) and phlegm and blood stasis syndrome (PBSS). 100 hospitalized patients with CHD with Qi deficiency and blood stasis syndrome (QDBSS) were rolled into the experimental (Exp) group (routine nursing intervention) and control (Ctrl) group (TCM nursing intervention, syndrome differentiation nursing), with 50 patients in each group. They underwent the intracoronary ultrasound imaging scanning. The results showed that after intervention, the plaque load (45.08 ± 6.02%), plaque eccentricity index (0.47 ± 0.08%), vascular remodeling index (0.53 ± 0.11%), and vascular external elastic membrane area (8.67 ± 3.06 mm^2^) of the Exp group were notably inferior to those of the Ctrl group (60.22 ± 5.82%, 0.59 ± 0.08%, 0.71 ± 0.09%, and 10.56 ± 2.31 mm^2^). The total effective rate in the Exp group (88%) was greatly superior to that of the Ctrl group (68%). In terms of TCM symptom scores, the TCM symptom scores of chest pain, chest tightness, and shortness of breath in the Exp group after intervention (1.07 ± 0.21 points, 0.75 ± 0.27 points, and 0.58 ± 0.12 points) were notably inferior to those in the Ctrl group (1.62 ± 0.28 points, 1.03 ± 0.21 points, and 0.79 ± 0.14 points). In the Exp group, after intervention, the degree of physical activity limitation (67.05 ± 5.08 points), the stable state of angina pectoris (65.28 ± 3.76 points), the frequency of angina pectoris attack (85.92 ± 2.97 points), the degree of treatment satisfaction (75.39 ± 5.94 points), the cognition score of disease (63.56 ± 5.84 points), the levels of triglyceride (1.27 ± 0.41 mmol/L), and total cholesterol (2.24 ± 0.41 mmol/L) were remarkably inferior to the Ctrl group (52.97 ± 4.31 points, 50.77 ± 4.69 points, 71.36 ± 3.77 points, 64.08 ± 5.64 points, 51.77 ± 6.33 points, 2.09 ± 0.57 mmol/L, and 3.06 ± 0.84 mmol/L) (*P* < 0.05). It suggested that intracoronary ultrasound imaging can clearly display the coronary plaques of patients and accurately evaluate the clinical efficacy of patients with CHD. The TCM nursing program can greatly improve the angina symptoms and quality of life of patients with CHD and PBSS, reduce blood lipid levels, and effectively improve the clinical efficacy of patients.

## 1. Introduction

Coronary artery disease (CHD), whose full name is coronary atherosclerotic heart disease, is caused by myocardial ischemia and hypoxia caused by coronary artery sclerosis. It is more common in middle-aged and elderly people, and its incidence increases with age [1, 2]. Many people have no obvious symptoms on weekdays but often suffer from myocardial ischemia. If they feel precardiac discomfort or fatigue, they must go to the hospital for electrocardiogram examination to diagnose and prevent it as soon as possible [3]. The current clinical treatment methods are drug therapy and interventional therapy [4–6]. In terms of drugs, calcium channel blockers, nitric lipids, and conversion enzyme inhibitors are usually selected. For patients with rapid heart rate, *β*-blockers, aspirin, or antiplatelet drugs can be used to prevent thrombosis. For patients with heart failure and arrhythmia, corresponding corrective treatment should be added, and coronary angioplasty and cardiac bypass surgery should be considered if the symptoms continue to worsen [7].

In addition to drug treatment and surgical treatment, modern medicine also pays attention to nursing interventions for patients. The occurrence of CHD is related to nature, society, and individual lifestyle [8]. In recent years, with the improvement of social economy and people's living standards, factors such as tobacco and alcohol, high-fat and high-salt diet, and reduced physical activity will greatly increase the incidence of CHD. At present, the main syndromes of CHD are Qi deficiency, blood stasis, phlegm turbidity, and phlegm-stasis [9, 10]. According to traditional Chinese medicine (TCM), CHD belongs to chest pain and heartache. The pathogenesis is mostly due to various factors such as the invasion of cold pathogens, emotional disorders, aging and physical weakness, or improper diet. Therefore, TCM nursing is often based on the basic principles of first protecting vitality, regulating Qi and removing blood stasis, maintaining a happy mood, and maintaining liver balance [11, 12].

At present, imaging techniques are mostly used for the diagnosis of CHD. Magnetic resonance imaging (MRI) is one of the common methods for diagnosing diseases in medical clinics. It can be used to examine diseases such as cardiovascular system, nervous system lesions, and thoracic lesions. It has high diagnostic accuracy but is expensive [13–15]. Echocardiography can clearly display the structure and movement of the heart, blood flow velocity, etc., and record the images of sound waves that are transmitted to the heart and return. It has the advantages of low cost and simple operation [16]. Coronary angiography (CAG) is the current gold standard for diagnosing CHD. It is characterized by obtaining the most intuitive imaging results in a relatively short period of time, but it can only reflect the outline of the lumen rather than the atherosclerotic plaque itself. Therefore, there are considerable limitations for the treatment program based on it [17, 18]. Intracoronary ultrasound is a new diagnostic method that combines noninvasive ultrasound and invasive catheter technology. It can not only quantitatively measure and analyze the diameter and degree of stenosis of blood vessels but also clarify the shape, nature, and distribution of coronary lesions, observe the progression and regression of coronary atherosclerosis, and assess the tension and compliance of blood vessel walls, showing high application value [19].

Therefore, a total of 100 inpatients with QDBSS of CHD were selected as the research subjects. The Ctrl group adopted conventional nursing measures and the Exp group adopted TCM nursing intervention based on that of the Ctrl group. The intravascular ultrasound imaging technology was used as an evaluation method. Imaging indexes (plaque burden, plaque eccentricity index, vascular remodeling index, and external elastic membrane area), total response rate, angina pectoris scale score, TCM syndrome score, and blood lipid level were used as evaluation indexes, to discuss the clinical efficacy of TCM nursing intervention program based on coronary ultrasound imaging in patients with phlegm-stasis syndrome of CHD, aiming to provide effective treatment and nursing ideas for patients with phlegm-stasis syndrome of CHD.

## 2. Materials and Methods

### 2.1. Subjects

In this study, 100 inpatients with CHD and QDBSS admitted to the hospital from November 10, 2020, to February 5, 2022, were recruited, including 63 males and 37 females. All patients were randomly assigned into the experimental (Exp) group (50 cases) and the control (Ctrl) group (50 cases). Subjects in the Ctrl group used routine nursing intervention program and intervention time for patients was from admission to discharge. The Exp group received conventional nursing combined with TCM nursing intervention program, and syndrome differentiation nursing was implemented. This study had been approved by ethics committee of hospital, and the patients and their families were informed and signed the informed consent.

#### 2.1.1. Inclusion Criteria

The inclusion criteria are as follows: patients over 35 years old; patients who can cooperate with follow-up; patients with complete basic information of the case; patients with clinical manifestations of chest pain and chest tightness, palpitations, shortness of breath, mental fatigue, and purple complexion dark, etc.; and patients who volunteered to participate in the experiment.

#### 2.1.2. Exclusion Criteria

The exclusion criteria are as follows: patients with severe heart failure; patients with mental disorders and unable to communicate normally; pregnant or breastfeeding women; patients with drug allergies; and patients who had been treated with drugs in the past six months.

### 2.2. Nursing Program

The specific nursing procedures in the Ctrl group were as follows. (I) First, it should ensure that the patient's ward is in good hygiene, with sufficient light, humidity, and temperature, and pay attention to regular disinfection. (II) It should assess the patient's pain situation, assist the patient to present an appropriate posture, monitor the changes of the patient's vital characteristics in real time, and pay attention to appease the patient's anxiety and tension. (III) It had to be cautious about the use of drugs, such as the use of nitrates to observe the patient's blood pressure level and monitor the patient's liver function if other statins were adopted. (IV) It should guide patients to have a healthy diet and quit smoking. Bad habits such as alcoholism and overeating.

The specific operations in the Exp group were as follows. (I) Real-time attention and assessment of the patient's chest pain. If the patient had symptoms such as aggravation of pain, sweating, and cold limbs, emergency treatment was required in time, the patient was given complete bed rest and oxygen support was given. (II) Pay attention to monitoring the patient's heart rate, systolic blood pressure, diastolic blood pressure, respiratory rate, and other vital characteristics, help the patient to adopt the most appropriate body position, and perform electrocardiogram examination and timely symptomatic treatment. (III) Explain the harm caused by constipation to the patient, instruct the patients to drink more hot water, eat more cellulose-rich fruits and vegetables, and nondiabetic patients can also drink 15 mL of honey water every day. (IV) Intervene the patient's sleep situation. If the patient often suffered from insomnia, it was necessary to reduce the redundant operations during naps and late nights, and play soft music in the ward. (V) A scientific and reasonable dietary plan needed to be formulated in response to the patient's dietary problems. CHD patients needed tonic food for promoting blood circulation and removing blood stasis, such as chicken, beef, yam, and jujube. Chinese medicine diet recommended peach kernel porridge (15 g peach kernel, 45 g japonica rice, first peel the peach kernel, grind it, boil the juice, and make porridge with the japonica rice), once a week. (VI) Provide emotional nursing for the anxiety and fear of the patient, communicate with the patient more, and use the method of transference, such as music therapy, to divert the patient's attention.

### 2.3. The Intracoronary Ultrasound Imaging Examination

First, CAG was performed, and the patient's femoral artery was used as the puncture point, and local anesthesia was administered. With the help of digital subtraction angiography X-ray machine, the catheter was sent into the puncture site, the contrast agent was infused, and finally, the stenosis degree and lesion area of the culprit vessel were measured. Then, on the basis of CAG, the ultrasound catheter was sent into the puncture site, the guide wire was withdrawn, and low molecular weight heparin was given for anticoagulation. Then, the ultrasound catheter was slowly withdrawn, and ultrasound imaging was performed during this process. Finally, PB, EI, EEMA, and vascular RI of diseased vessels were calculated according to the ultrasound images.

#### 2.3.1. Plaque Burden (PB)

Plaque cross-sectional area/external elastic membrane cross-sectional area represented the proportion of plaque to external elastic membrane area.

#### 2.3.2. Plaque Eccentricity Index (EI)

(Maximum plaque thickness-minimum plaque thickness)/maximum plaque thickness. EI < 0.5 referred to centripetal plaque, and EI ≥ 0.5 referred to eccentric plaque. The higher the EI value was, the more obvious the degree of plaque eccentricity was.

#### 2.3.3. External Elastic Membrane Area (EEM)

The inner edge of the outer membrane was recorded manually and measured by a computer automatic edge measurement system.

#### 2.3.4. Vascular Remodeling Index (RI)

Mean cross-sectional area of external elastic membrane at the lesion/mean cross-sectional area of reference segment. If RI > 1.05, positive reconstruction was considered. If RI < 0.95, inverse reconstruction was considered.

### 2.4. Observation Indicators

The gender, age, height, weight, disease duration, comorbidities, and stability angina pectoris classification under Canadian Cardiovascular Society (CCS) of patients were collected. The frequency of angina pectoris and degree of angina pectoris of the patients were recorded. The data of patients before and after nursing intervention and two weeks after discharge in outpatient follow-up were recorded. The Seattle Angina-pectoris Scale (SAQ) was adopted to evaluate the patients' quality of life, including five items: degree of physical activity limitation, stable state of angina pectoris, frequency of angina pectoris, treatment satisfaction, and disease awareness. In addition, the satisfaction with nursing interventions was assessed using the Mueller/McCloskey Nurse Job Satisfaction Scale. Before and after nursing intervention, serum lipid levels (triglyceride, total cholesterol, and low-density lipoprotein) in fasting state were detected in the morning.

### 2.5. Statistical Processing

SPSS 26.0 was employed for data process. Measurement data were denoted as mean ± standard deviation ($\bar{x}$ ± *s*). Counting data were statistically inferred by *χ*^2^ test. *P* < 0.05 was statistically considerable.

## 3. Results

### 3.1. General Data

The general data of the patients in the Exp group and Ctrl group were compared (Figure 1). The number of males and females, age distribution, height, weight, comorbidities (hypertension, hyperlipidemia, and diabetes), CCS stability angina pectoris grade, and average course of disease were not greatly different between the groups (*P* > 0.05).

### 3.2. Case Analysis

Figure 2 shows intracoronary ultrasound images of a 62-year-old male patient in the Exp group before and after intervention, and CAG showed simultaneous closure of the anterior descending branch. The length of the block was about 21 mm. The patient had anterior descending artery occlusion combined with ischemia, suggesting viable myocardium. There was no residual complete occlusion of the anterior descending artery, and the route of the occlusive end was unclear. According to the image, the diameter and effective lumen area of the patient after treatment combined with TCM nursing intervention were greatly smaller than before treatment.

### 3.3. Comparison of the Curative Effect between the Two Groups of Patients

In Figure 3, in the Exp group, 17 cases were markedly effective, 27 were effective, and 6 were ineffective; while in the Ctrl group, 11 were markedly effective, 23 were effective, and 16 were ineffective. The analysis showed that the total effective rate of patients in the Exp group (88%) was greatly superior to the Ctrl group (68%) (*P* < 0.05).

### 3.4. TCM Symptom Score before and after Intervention

In Figure 4, no evident difference was found in the TCM symptom score of chest pain, chest tightness, and shortness of breath between groups before intervention (*P* > 0.05). The TCM symptom scores of chest pain, chest tightness, and shortness of breath in the two groups after intervention were notably inferior to those before intervention (*P* < 0.05). The abovementioned TCM symptom scores in the Exp group after intervention were remarkably inferior to those of the Ctrl group (*P* < 0.05).

### 3.5. Comparison of Angina Pectoris Scale Scores before and after Intervention

In Figure 5, there was no evident difference in the degree of physical activity limitation, stable state of angina pectoris, frequency of angina pectoris, treatment satisfaction, and disease awareness score between groups before intervention (*P* > 0.05). The degree of physical activity limitation, stable state of angina pectoris, frequency of angina pectoris, treatment satisfaction, and disease awareness score in the two groups after intervention were notably inferior to those before intervention (*P* < 0.05), while those in the Exp group after intervention were remarkably inferior to the Ctrl group, with statistical significance (*P* < 0.05).

### 3.6. Intracoronary Ultrasound Indexes of Patients before and after Intervention

In Figure 6, there was no evident difference in the PB, plaque EI, vascular RI, and EEMA between groups before intervention (*P* > 0.05). The PB, plaque EI, vascular RI, and EEMA after intervention in the two groups were notably inferior to those before intervention (*P* < 0.05). After intervention, the PB, plaque EI, vascular RI, and EEMA in the Exp group were remarkably inferior to the Ctrl group (*P* < 0.05).

### 3.7. Blood Lipid Levels before and after Intervention

In Figure 7, no evident difference was indicated in the TG and TC levels between groups before intervention (*P* > 0.05). The TG and TC of the two groups of patients after intervention were notably inferior to those before intervention (*P* < 0.05). After intervention, the TG and TC in the Exp group were remarkably inferior to those in the Ctrl group (*P* < 0.05). In addition, there was no evident difference in the LDL level between groups before and after the intervention (*P* > 0.05).

### 3.8. Nursing Satisfaction

In Figure 8, the satisfaction score of the patients in the Exp group was 28.71 ± 4.02 points; while the satisfaction score of the patients in the Ctrl group was 21.53 ± 3.29 points. Among them, the satisfaction score of patients in the Exp group was greatly superior to the Ctrl group (*P* < 0.05).

## 4. Discussion

CHD is an aging disease with extremely high morbidity, disability, and fatality rate, which brings huge economic burden and mental pressure to people's daily life and society. In recent years, there has been a trend toward younger age. Therefore, seeking better diagnosis and treatment methods is also the focus of current research [20]. Interventional CAG is a common method for diagnosing CHD, but its diagnostic accuracy is not high, and it is prone to misdiagnosis and misdiagnosis [21].

Therefore, this work selected 100 inpatients with CHD and QDBSS as the research objects. All patients were divided into an Exp group (routine nursing intervention program) and a Ctrl group (the TCM nursing intervention program on the basis of routine nursing to carry out syndrome differentiation nursing), with 50 cases in each group. Intracoronary ultrasound imaging scans before and after concurrent treatment. First, the basic data were compared, and it was found that there were no statistical differences in the number of males and females, age distribution, height, weight, comorbidities (hypertension, hyperlipidemia, and diabetes), CCS stability angina pectoris classification, and average course of disease between groups of patients showed no great significance (*P* > 0.05), which provided conditions for the follow-up case-control study. Then, the intracoronary ultrasound imaging performance of a 62-year-old male patient before and after intervention was analyzed. Before treatment, CAG showed that the patient's anterior descending artery was closed together with ischemia symptoms, and the route of the occlusion end was unclear. The diameter and effective lumen area of patients after treatment were greatly smaller than those before treatment, which indicated that intracoronary ultrasound imaging can accurately assess the clinical efficacy of CHD patients. From the quantitative indexes of intracoronary ultrasound, the PB, plaque EI, vascular RI, and EEMA of the Exp group after intervention were notably inferior to those of the Ctrl group (*P* < 0.05). This confirms the considerable effect of TCM care on CHD patients from an imaging point of view.

In terms of clinical efficacy, it was found in this work that the total effective rate of patients in the Exp group (88%) was greatly higher versus the Ctrl group (68%) (*P* < 0.05). Such result is similar to the findings of Richards et al. [22], which show that the TCM nursing regimen can notably enhance the symptoms of angina pectoris in patients with CHD and PBSS compared with the routine nursing regimen, with a considerable effect. In terms of TCM symptom score, this work revealed that the TCM symptom score of chest pain, chest tightness, and shortness of breath in Exp group after intervention was notably inferior to that in Ctrl group (*P* < 0.05). The TCM nursing program pays attention to dialectical nursing, and can provide corresponding nursing intervention measures according to the individual situation of the patient, which can be supplemented by the technical treatment of TCM characteristics, which shows that the TCM nursing program has high clinical application value [23]. After intervention, the degree of physical activity limitation, stable state of angina pectoris, frequency of angina pectoris, treatment satisfaction, and disease awareness score in Exp group were remarkably inferior to Ctrl group, showing statistically evident differences (*P* < 0.05). This shows that the TCM nursing program can remarkably alleviate the adverse physiological and psychological changes caused by the progression of the disease, relieve the physical and mental pain of the patient, and improve the quality of life. The TG and TC in the Exp group after intervention were remarkably inferior to the Ctrl group (*P* < 0.05). TG and TC are two of the four indicators of blood lipids. Elevated TG and TC levels can cause cardiovascular and cerebrovascular damage, accelerate atherosclerosis and plaque formation, and increase the occurrence of cardiovascular events such as myocardial infarction and cerebral infarction [24]. Thus, the results indicate that the TCM care regimen can effectively reduce the patient's blood lipid level and reduce the risk of disease deterioration in CHD patients.

## 5. Conclusion

In this study, different nursing intervention schemes were adopted for patients in the Exp group and Ctrl group, and coronary ultrasound scan was performed before and after treatment. The results found that intravascular ultrasound can clearly display the coronary plaque and accurately evaluate the clinical efficacy of patients with CHD. Compared with conventional nursing, TCM nursing program can greatly improve angina pectoris symptom and life quality of patients with phlegm-stasis syndrome of CHD, reduce blood lipid level, and effectively improve clinical efficacy. Limited by time and region, this study only included cases of phlegm-stasis syndrome of CHD admitted to hospital. The sample size was small and the study was not comprehensive enough. Moreover, subjective questionnaires were mostly used as evaluation criteria, which may have some influence on the results. In the future, the scope of the study will be expanded to include CHD patients from different regions and hospitals and patients of different TCM syndromes for further analysis. In conclusion, this study provides a reference for the combined application of imaging technology and TCM nursing intervention in the clinical treatment of CHD.

## Figures and Tables

**Figure 1:** General data of the two groups. A∼F shows the comparison of the number of males and females, height and weight, age distribution, comorbidities, CCS stability angina pectoris grade, and average course of disease, respectively.

**Figure 2:** Intracoronary ultrasound imaging of a male patient before and after treatment (62 years old, admitted to the hospital for CHD unstable angina pectoris). A–C shows the intracoronary ultrasound imaging performance of the patient before treatment, the anterior descending branch was occluded with ischemia symptoms; D–E shows the intracoronary ultrasound imaging performance of the patient before and after treatment, occlusive coronary artery was successfully opened and the clinical effect was definite.

**Figure 3:** Clinical efficacies between groups of patients. (a) shows the numbers of markedly effective, effective, and ineffective cases; (b) shows the total effective rate. ^*∗*^Compared with the Ctrl group, *P* < 0.05.

**Figure 4:** TCM symptom scores before and after intervention. (a) refers to chest pain; (b) refers to chest tightness; and (c) represents shortness of breath. ^*∗*^Compared with that before intervention, *P* < 0.05; ^#^compared with the Ctrl group, *P* < 0.05.

**Figure 5:** Angina pectoris scale scores before and after intervention in the two groups A–E shows the degree of physical activity limitation, stable state of angina pectoris, frequency of angina pectoris, treatment satisfaction, and disease awareness, respectively. ^*∗*^Compared with that before intervention, *P* < 0.05; ^#^compared with the Ctrl group, *P* < 0.05.

**Figure 6:** Comparison of intracoronary ultrasound indexes before and after intervention in two groups. A–D are the comparisons of PB, plaque EI, vascular RI, and EEMA, respectively. ^*∗*^Compared with that before intervention, *P* < 0.05; ^#^compared with the Ctrl group, *P* < 0.05.

**Figure 7:** Blood lipid levels in the two groups before and after intervention. A–C shows the comparison on TG, TC, and LDL, respectively. ^#^Compared with the Ctrl group, *P* < 0.05.

**Figure 8:** Comparison of the satisfaction of patients with nursing. ^*∗*^Compared with the Ctrl group, *P* < 0.05.

## Data Availability

The data used to support the findings of this study are available from the corresponding author upon request.

## References

[1] Wirtz P. H., Von Känel R. (2017). Psychological stress, inflammation, and coronary heart disease. *Current Cardiology Reports*.

[2] Tian Y., Deng P., Li B. (2019). Treatment models of cardiac rehabilitation in patients with coronary heart disease and related factors affecting patient compliance. *Reviews in Cardiovascular Medicine*.

[3] Katta N., Loethen T., Lavie C. J., Alpert M. A. (2021). Obesity and coronary heart disease: epidemiology, pathology, and coronary artery imaging. *Current Problems in Cardiology*.

[4] Dong Y., Chen H., Gao J., Liu Y., Li J., Wang J. (2019). Molecular machinery and interplay of apoptosis and autophagy in coronary heart disease. *Journal of Molecular and Cellular Cardiology*.

[5] Zhao R., Sun K., Zhao R. (2018). Inflammatory biomarkers of coronary heart disease. *Frontiers in Bioscience*.

[6] De Hert M., Detraux J., Vancampfort D. (2018). The intriguing relationship between coronary heart disease and mental disorders. *Dialogues in Clinical Neuroscience*.

[7] Stewart R. A. H., Held C., Hadziosmanovic N. (2017). Physical activity and mortality in patients with stable coronary heart disease. *Journal of the American College of Cardiology*.

[8] Cybulska B., Kłosiewicz-Latoszek L. (2019). Landmark studies in coronary heart disease epidemiology. The framingham heart study after 70 years and the seven countries study after 60 years. *Kardiologia Polska*.

[9] Rush C. J., Berry C., Oldroyd K. G. (2021). Prevalence of coronary artery disease and coronary microvascular dysfunction in patients with heart failure with preserved ejection fraction. *JAMA Cardiol*.

[10] Walker S., Cox E., Rothwell B. (2021). Cost-effectiveness of cardiovascular imaging for stable coronary heart disease. *Heart*.

[11] Sperry B. W., Qarajeh R., Omer M. A. (2021). Influence of donor transmitted and rapidly progressive coronary vascular disease on long-term outcomes after heart transplantation: a contemporary intravascular ultrasound analysis. *Journal of Cardiac Failure*.

[12] Mondal P., Aljizeeri A., Small G. (2021). Coronary artery disease in patients with human immunodeficiency virus infection. *Journal of Nuclear Cardiology*.

[13] Xiao J., Lu Y., Yang X. (2020). Ultrasound detection of epicardial adipose tissue combined with ischemic modified albumin in the diagnosis of coronary heart disease. *The Heart Surgery Forum*.

[14] Monti C. B., Codari M., De Cecco C. N., Secchi F., Sardanelli F., Stillman A. E. (2020). Novel imaging biomarkers: epicardial adipose tissue evaluation. *British Journal of Radiology*.

[15] Hong M. K., Lee S. Y. (2021). Intravascular ultrasound for percutaneous coronary intervention: benefits and limitations. *JACC: Cardiovascular Interventions*.

[16] Wang X., Yu D., Wang J., Huang J., Li W. (2021). Analysis of coronary artery lesion degree and related risk factors in patients with coronary heart disease based on computer-aided diagnosis of coronary angiography. *Computational and Mathematical Methods in Medicine*.

[17] Cobo D. L., Batigalia F., Croti U. A., Sciarra A. M. P., Foss M. H. D., Cobo R. G. F. (2021). Fístula da Artéria Coronária: a. *Arquivos Brasileiros de Cardiologia*.

[18] de la Torre Hernandez J. M. (2021). Imaging and physiology get along in the left main coronary artey disease: the case for intravascular ultrasound and instantaneous wave-free ratio. *Circulation: Cardiovascular Interventions*.

[19] Lin C., Xie C., Chen M., Gao H., Zhang G. (2021). Effect of continuous traditional Chinese medicine nursing on patients with coronary heart disease. *Am J Transl Res*.

[20] Houston M. (2018). The role of noninvasive cardiovascular testing, applied clinical nutrition and nutritional supplements in the prevention and treatment of coronary heart disease. *Ther Adv Cardiovasc Dis*.

[21] Lao X. Q., Liu X., Deng H. B. (2018). Sleep quality, sleep duration, and the risk of coronary heart disease: a prospective cohort study with 60,586 adults. *Journal of Clinical Sleep Medicine*.

[22] Richards S. H., Anderson L., Jenkinson C. E. (2018). Psychological interventions for coronary heart disease: cochrane systematic review and meta-analysis. *European Journal of Preventive Cardiology*.

[23] Xin G. J., Fu J. H., Li L. (2020). Research progress of traditional Chinese medicine in regulating autophagy and ischemic heart disease. *Zhongguo Zhong Yao Za Zhi*.

[24] Liu T., Chan A. W. K., Taylor-Piliae R. E., Choi K. C., Chair S. Y. (2021). Psychometric properties of the translated tai chi exercise self-efficacy scale for Chinese adults with coronary heart disease or risk factors. *International Journal of Environmental Research and Public Health*.

